The article "Altered Expression of Survivin Variants S-2B and S-WT in Breast Cancer Is Related to Adipokine Expression" was published in 2022. Journal: J Oncol.

# Altered Expression of Survivin Variants *S-2B* and *S-WT* in Breast Cancer Is Related to Adipokine Expression

**DOI:** 10.1155/2022/7398444

**Published:** 2022-03-16

**Authors:** Dora Maria Cedano-Prieto, Fernando Bergez-Hernandez, Emir Adolfo Leal-Leon, Noemi Garcia-Magallanes, Fred Luque-Ortega, Veronica Picos-Cardenas, Edna Guerrero-Arambula, Bricia Gutierrez-Zepeda, Enrique Romo-Martinez, Eliakym Arambula-Meraz

**Affiliations:** ^1^Laboratorio de Genética y Biología Molecular, Facultad de Ciencias Químico Biológicas, Universidad Autónoma de Sinaloa, Culiacán 80010, Mexico; ^2^Posgrado en Ciencias Biomédicas, Facultad de Ciencias Químico Biológicas, Universidad Autónoma de Sinaloa, Culiacán 80010, Mexico; ^3^Laboratorio de Biomedicina y Biología Molecular, Unidad Académica de Ingeniería en Biotecnología, Universidad Politécnica de Sinaloa, Mazatlán 82199, Mexico; ^4^Laboratorio de Ciencias Básicas, Facultad de Odontología, Universidad Autónoma de Sinaloa, Culiacán 80010, Mexico; ^5^Laboratorio de Genética, Facultad de Medicina, Universidad Autónoma de Sinaloa, Culiacán 80119, Mexico

## Abstract

Breast cancer (BCa) is one of the leading causes of death in women with these types of malignancies. Early detection is pivotal to improve prognosis and reduce mortality. Several proteins and genes have been proposed as biomarkers for cancer; however, further studies are required before a molecule is accepted as a definitive biomarker. This study was aimed at investigating the expression of survivin variants *S-WT*, *S-2B*, and *S-ΔEx3*, as well as adipokines *LEP* and *ADIPOQ* in breast cancer. Breast samples were obtained from patients with (*n* = 27) and without (*n* = 20) BCa, and relative gene expression was assessed by RT-qPCR. *S-WT* and *S-2B* showed a significant increase in BCa samples (*p* = 0.005 and *p* = 0.001, respectively) and in high-aggressiveness BCa (*p* = 0.026 and *p* = 0.037, respectively). Despite *S-ΔEx3* expression remained globally unchanged, when dividing BCa samples according to the stage, this gene showed a significant tendency to increase towards more advanced stages, and the exact opposite effect was observed for *LEP*. Furthermore, *LEP* expression showed a negative correlation with *S-2B* (*p* = 0.005) and *S-WT* (*p* = 0.011), and in the same manner, *ADIPOQ* was negatively related with these two survivin variants (*p* = 0.001 and *p* = 0.005, respectively). Interestingly, *S-ΔEx3* expression appears unaffected by *LEP* and *ADIPOQ* expressions. Our results highlight the importance of investigating specific variants of a given gene, as sequence variation may grant different correlation with other important structures and diseases.

The article "Altered Expression of Survivin Variants S-2B and S-WT in Breast Cancer Is Related to Adipokine Expression" was published in 2022. Journal: J Oncol.

## 1. Introduction

Breast cancer (BCa) is the second cause of cancer worldwide and the first type of cancer diagnosed in women. It also represents a public health problem as is the cancer with the highest mortality in women [1]. The high incidence of BCa originates as a consequence of deficient early detection and adequate diagnosis [2]. To address this problem, it is necessary to understand the molecular characteristics of the disease. In this matter, several biomarkers of single- or multigene signatures have been approved for clinical use in BCa prognosis. Currently, a large number of molecular biomarkers are being studied in an effort to facilitate the diagnosis, early detection, accurate prediction of metastatic behaviors, and selection of therapy [3].

Over the years, various studies have shown an existing association between an elevated *BIRC5* expression and BCa [4–6]. This gene codes for the survivin protein, which plays a dual role in regulating cell division and apoptosis [7, 8]. The expression of *BIRC5* elevates during fetal development, and the same occurs in most tumors, but it is otherwise low in adult tissues [9]. Interestingly, depending on the different junction, *BIRC5* encodes three different mRNAs that share their names with the proteins that they produce: *S-WT* (Survivin-WT or S-WT), *S-2B* (Survivin-2B or S-2B), and *S-ΔEx3* (Survivin-*Δ*Ex3 or S-*Δ*Ex3). It was suggested that *S-WT* and *S-ΔEx3* expressions are associated with a poor BCa prognosis, by acting as apoptosis inhibitors. On the contrary, S-2B protein may possess a proapoptotic role as this isoform dimerizes with S-WT protein causing its loss of function [10, 11]. It is suggested that survivin isoforms may be related to clinicopathological characteristics such as cancer stage and estrogen receptor status, and that they may have prognostic significance [5, 12, 13]. Specifically, *S-WT* and *S-2B* have been associated with tumor stage and estrogen receptors, where high *S-2B* expression is associated with a better prognosis. On the other side, *S-ΔEx3* is associated with tumor malignancy degree [4–6, 14]. These findings highlight the importance of investigating the survivin variants, which roles in BCa remain poorly understood, despite the interesting results that have been reported [4].

In this same context, the roles of adipokines on BCa development have been studied as well. These hormones are primarily expressed in adipose tissue. Given that a woman breast is composed of more than 80% of this tissue [15], it is not surprising that adipokines such as leptin and adiponectin are related to BCa development [16]. Leptin acts as a central mediator in the regulation of appetite and energy homeostasis [17]. It has also shown the ability to promote growth, migration, invasion, and angiogenesis of tumor cells, and when its circulating levels are elevated, the risk of developing BCa is increased [18–20]. On the other hand, adiponectin is the most abundant adipokine. It possesses anti-inflammatory, antiteratogenic, and antitumor effects [21, 22]. However, the opposite effect has been observed in BCa, where it increases cell proliferation in estrogen receptor-positive cells, showing a dichotomous effect on BCa growth depending on estrogen receptor status [23]. Likewise, results evidence that adiponectin may be involved in early stages of metastasis progression [24].

The article "Altered Expression of Survivin Variants S-2B and S-WT in Breast Cancer Is Related to Adipokine Expression" was published in 2022. Journal: J Oncol.

Therefore, bringing into the light, the expression of genes in charge of encoding proteins related to BCa development is decisive to improve molecular prognosis, diagnosis, and treatment of this pathology. Thus, this study was aimed at analyzing the expression of genes *S-WT*, *S-2B*, *S-ΔEx3*, *LEP* (leptin), and *ADIPOQ* (adiponectin), as well as their correlations.

## 2. Materials and Methods

### 2.1. Tissue Samples

Tissue samples were obtained through breast biopsy. Our study group consisted of 47 samples divided into two groups, 27 from patients diagnosed with BCa, and 20 from patients diagnosed with benign breast tumors (BBT). As established by the inclusion criteria, patients were women older than 18 years, with diagnosis for BCa or BBT confirmed by histopathology, neither receiving chemotherapy nor radiotherapy, and presenting no other type of cancer. All patients were recruited from the Instituto de Cancerologia de Sinaloa (ICS) located in Sinaloa, Mexico, from February 2017 to February 2018. Clinicopathological data were collected through direct questionnaire and hospital database. Patients granted approval by signing an informed consent that was previously reviewed and approved by the Ethics and Research Committee of the ICS.

### 2.2. RNA Extraction

Total RNA was isolated using the TRIzol LS (Ambion®, Austin, USA) method according to manufacturer instructions. Isolated RNA concentration was measured with assistance of a GENESYS 10S UV-Vis Spectrophotometer (Thermo Scientific™).

### 2.3. Relative Gene Expression

Reverse transcription (RT) was performed from 10 ng of total RNA with the ImProm-II™ Reverse Transcriptase Kit (Promega Corporation, Madison, WI, USA) and oligo dT. Quantitative estimations of *S-WT*, *S-2B*, *S-ΔEx3*, *LEP*, and *ADIPOQ* transcripts were performed by real-time PCR (RT-qPCR) method using TaqMan® Assays (Applied Biosystems) on a StepOnePlus™ Real-Time PCR system (Applied Biosystems). *Beta-actin* (*Act-®*) was used as reference gene to normalize the expression of our genes of interest. Reaction conditions were as described in Arámbula-Meraz et al. [25]. All samples were assessed in technical duplicates. To quantify relative gene expression, we used the method of Livak and Schmittgen [26].

The article "Altered Expression of Survivin Variants S-2B and S-WT in Breast Cancer Is Related to Adipokine Expression" was published in 2022. Journal: J Oncol.

### 2.4. Statistical and Correlational Analysis

The Student's *t*-test and Mann–Whitney *U* test (when appropriate) were used to compare differences between continuous variables. Pearson's *χ*^2^ test was used to compare the differences between dichotomous variables. Pearson and Spearman tests (when appropriate) were used to calculate the correlation coefficient between variables: *S-WT*, *S-2B*, *S-ΔEx3*, *LEP*, and *ADIPOQ* expression, patient age, body mass index, age of menarche, pregnancies, tumor stage, and hormone receptor percentages. All variables were contrasted to each other. The Statistical Package for the Social Sciences (SPSS, Inc., Chicago, IL,) version 20 software was used for all statistical calculations. Results with a *p* value < 0.05 were considered statistically significant.

## 3. Results and Discussion

### 3.1. Results

#### 3.1.1. Clinicopathological Characteristics

BCa and BBT patients had average ages of 55.37 ± 14.45 and 40.75 ± 7.95 years (*p* = 0.001), respectively. Evaluation of body mass index (BMI) yielded averages of 27.66 ± 14.18 and 30.06 ± 6.13 kg/m^2^ for BCa and BBT patients, respectively; accordingly to these results, no statistical significance was found between groups (*p* = 0.140). Concerning the age of menarche, we found that the average ages in BCa and BBT patients were 13.41 ± 1.58 and 12.85 ± 1.46 years, respectively; thus, statistical difference between groups was not observed (*p* = 0.223) (Table 1).

Analyzing menopause onset, BCa patients showed an average age of 47.43 ± 4.05 years and BBT patients an average age of 39.67 ± 6.12 years (*p* = 0.010). When evaluating the number of pregnancies, we found that the BCa group had a higher number of pregnancies (approximately 4) when compared with the BBT group (approximately 2); however, we found no statistical difference (*p* = 0.138). Nevertheless, when analyzing the average age of first pregnancy, BCa patients presented an average age of 30.41 ± 6.40 years and BBT patients an average age of 20.44 ± 4.29 years, resulting in a significant difference between groups (*p* = 0.001) (Table 1). When performing a Spearman correlation test, we observed that there was a relationship between the number of pregnancies and the age of first pregnancy (*p* = 0.032, *ρ* = 0.413). Moreover, analyzing the age of menarche and age of the first pregnancy, we observed a statistically significant relationship (*p* = 0.026, *ρ* = 0.429). Lastly, regarding BCa stage, we found that 11.12% were classified as IA, 33.33% as IIA, 22.22% as IIB, 14.81% as IIIA, and 18.52% as IIIB (Table 2).

The article "Altered Expression of Survivin Variants S-2B and S-WT in Breast Cancer Is Related to Adipokine Expression" was published in 2022. Journal: J Oncol.

#### 3.1.2. Relative Gene Expression

During the PCR procedure, several BBT and BCa samples expressed an unquantifiable gene expression; this was the case for all five genes, although, depending on the specific gene, a different number of samples presented this behavior. For the BBT group, we quantify gene expression for every gene from all samples (*n* = 20, for each gene), except for *S-ΔEX3* (*n* = 8). For the BCa group, we obtained *n* = 25, 20, 15, 25, and 25 for *S-WT*, *S-2B*, *S-ΔEX3*, *LEP*, and *ADIPOQ*, respectively. BCa samples and samples that showed quantifiable gene levels were divided according to cancer stage (Table 2).

For *LEP* and *ADIPOQ*, we found no significant differences in expression between BCa and BBT patients (*p* = 0.513 and *p* = 0.235, respectively), as shown in Figure 1. However, *S-2B* and *S-WT* showed a 13.01-fold and an 8.59-fold overexpression, respectively, in BCa patients when compared with BBT patients (*p* = 0.001 and *p* = 0.005, respectively) (Figure 1). Furthermore, *LEP* and *S-ΔEx3* expressions were also statistically different among cancer stages. In the case of *LEP*, we observed a significant difference between the stages IA and IIIA and IA and IIIB, as well as IIA and IIIB (*p* = 0.045, *p* = 0.003, and *p* = 0.032, respectively). Concerning *S-ΔEx3*, we found a significant difference between the stages IA and IIIA, IA and IIIB, and IIA and IIIA, as well as IIA and IIIB (*p* = 0.024, *p* = 0.022, and *p* = 0.023 and 0.028, respectively) (Figure 2).

Samples were also classified according to BCa subtype as described in Sandberg et al. [27]. Results showed that 18.51% of all BCa samples were classified as luminal A, 18.51% as luminal B, 33.33% as luminal HER2, 18.51% as HER2-enriched, and 11.11% as Basal-like (also known as TNBC, triple-negative breast cancer). We further grouped BCa subtypes according to aggressiveness, as low and high. Therefore, low-aggressiveness subtypes luminal A, B, and HER2 were merged into a group named “Luminal,” and high-aggressiveness subtypes HER2-enriched and Basal-like were combined into a group named “HER2-Basal” [28, 29]. When comparing these two groups, we observed a significant overexpression of *S-WT* and *S-2B* in the HER2-Basal group (*p* = 0.026 and *p* = 0.037, respectively) (Figure 3).

#### 3.1.3. Correlation Analysis

In BCa samples, this analysis demonstrated several correlations between different genes (Figure 4). We observed that *LEP* expression is related to the expression of *ADIPOQ*, *S-WT*, and *S-2B* (*p* = 0.001, *p* = 0.011, and *p* = 0.005, respectively) with correlation coefficients of 0.952, -0.511, and -0.578, respectively. Moreover, we found that *ADIPOQ* expression is negatively related to the expression of *S-WT* and *S-2B* (*p* = 0.005 and *p* = 0.001, respectively) with correlation coefficients of -0.551 and -0.645, respectively. A correlation (with coefficient of 0.817) between the expression of *S-WT* and *S-2B* (*p* = 0.001) was also observed. Lastly, it is important to remark that we did not observe correlations between *LEP* and *ADIPOQ* expressions with *S-ΔEx3* variant.

The article "Altered Expression of Survivin Variants S-2B and S-WT in Breast Cancer Is Related to Adipokine Expression" was published in 2022. Journal: J Oncol.

### 3.2. Discussion

Cancer is a multifactorial disease, and BCa is not an exception. Several risk factors have been associated with this disease over the last decades. In general, it is well recognized that hormones play an important role in BCa development [30]. These biomolecules are especially relevant for women. During her lifetime, a woman experiences different natural events that alter hormonal levels such as menarche, pregnancy, and menopause. Therefore, the age at which these alterations occur become key for BCa. Even though we found that the age of menarche had not a clear role, we observed an important impact of pregnancy and menopause. Results showed that the earlier in life these two events occur, the lower the risk of developing BCa. Moreover, aging is another natural event that has been deeply associated with breast cancer [31]. We observed a significant difference between the two groups, further supporting that BCa is associated with aging. However, natural processes are not the only risk factors; clinical conditions such as obesity have also been associated with BCa. In this matter, BMI is the gold standard to determine this condition. In our study, both groups exhibited similar BMI averages; interestingly and although barely, BBT patients presented an average BMI that classified them as an obese group, whereas BCa patients were classified as an overweighted group [32]. This demonstrates the important role of adipose tissue even at a benign stage.

Dysregulation of gene expression is a common event in breast cancer. Therefore, analysis of genes associated with cell survival may provide important information about the development and progression of this disease. *LEP* and *ADIPOQ* are two adipokines widely associated to BCa development; in adults, they are normally produced by subcutaneous adipocytes distributed through the entire body, and in consequence, they are deeply related to obesity as well. Proteins produced by these two genes, leptin and adiponectin, are well recognized by their proinflammatory and cell survival functions, as well as by their carcinogenic activities [21, 22]. The majority of studies have demonstrated that *LEP* and *ADIPOQ* expressions are diminished to a 30% in BCa tissue when compared to normal tissue adjacent to malignant tissue [33]. In our study, when comparing the expression between BCa and BBT groups, no significant differences were observed for *LEP* and *ADIPOQ*. This similar expression patterns in both groups suggest that the downregulation of these adipokines initiates prior to a malignant stage is reached. Importantly, we noticed that *LEP* presented a biphasic expression; this gene expression varied according to BCa stages. We observed a *LEP* overexpression in early stages (IA and IIA), with a sequential decrease towards more advanced stages. Previous reports have showed a similar behavior, finding that in high-grade tumors, there is a lower *LEP* expression when compared with low-grade tumors. It has been proposed that this occurs given the substitution of adipose tissue by cancerous epithelial cells; breast adipose tissue decreases as BCa progresses, thus, also explaining the *LEP* tendency to carry on decreasing from early to advanced stages [34, 35]. It is now known that *LEP* signaling promotes cell cycle and inhibits apoptosis via JAK2/STAT3 pathway and that survivin is a target gene for STAT3 in BCa cells [36, 37]. In the case of *ADIPOQ*, it has been observed that STAT3 is also a common downstream effector of adiponectin. Moreover, the promotion of tumor cell survival is partly mediated by activating STAT3 through survivin upregulation, and in this matter, *ADIPOQ* has been reported to decrease survivin transcription [38, 39].

The article "Altered Expression of Survivin Variants S-2B and S-WT in Breast Cancer Is Related to Adipokine Expression" was published in 2022. Journal: J Oncol.

On the other hand, the three protein isoforms of survivin have been attributed with regulation of cell proliferation and apoptosis [4–6]. Although elevated in cancer, survivin levels are either greatly diminished or null in normal adult breast tissue [40–42]; evaluating whether these levels remain low or absence during a benign stage, prior to malignant stages, or if they are elevated before the malignancy is developed, is of the most importance. To better understand this phenomenon, the expression of the three survivin variants (*S-WT*, *S-2B*, and *S-ΔEx3*) was quantified in BCa and BBT tissue samples. However, *S-WT*, *S-2B*, and *S-ΔEx3* variants were detected and quantified only in 91.33%, 74.07%, and 55.55% of all BCa samples, respectively. This apparent lack of detection is similar to that reported by Végran et al., where *S-WT* was detected in most samples, with the lowest detection percentage corresponding to *S-ΔEx3* [13]. When comparing relative expression between the two groups, we observed a significant *S-2B* and *S-WT* overexpression in BCa samples; however, *S-ΔEx3* expression remained statistically unchanged. Moreover, *S-2B* and *S-WT* were also statistically overexpressed in high-aggressiveness BCa samples. Similar to our results, Pavlidou et al. reported that *S-2B* and *S-WT* are the two main survivin variants overexpressed in BCa. Nevertheless, different types of cancer may present a distinct expression pattern, such is the case for oral cancer, where *S-WT* is the most overexpressed variant [4, 5, 43]. Furthermore, *S-2B* has been suggested as a biomarker and a novel therapeutic target due to its expression pattern and the possibility to detect it both in blood and tissue [13, 44]. This highlights the existence of specific gene expression patterns for each cancer type that we have yet to discover. Moreover, different BCa stages may present different gene expression as well, such is the case of the *S-ΔEx3* variant. *S-ΔEx3* was amplified in approximately 50% of all samples. It demonstrated similarly unquantifiable sample rates in the BCa and BBT groups; interestingly, it displays a positive relationship with cancer stage. Thus, as tumor advances in stages, *S-ΔEx3* expression increases. This agrees with various studies that have proved that this variant is mostly expressed and quantifiable in advanced stage tumors [5, 13].

The article "Altered Expression of Survivin Variants S-2B and S-WT in Breast Cancer Is Related to Adipokine Expression" was published in 2022. Journal: J Oncol.

Our results further support that *S-2B* is an interesting variant. We observed that *S-2B* expression relates to *LEP*, *ADIPOQ*, and *S-WT* expression. It was previously reported that *S-2B* expression is positively correlated with the *S-WT* expression in BCa [4, 45]. Although S-2B is considered a proapoptotic protein, its overexpression has been observed in advanced stage and androgen receptor-negative tumors, suggesting its potential usage as biomarker of aggressiveness in the absence of these receptors [4]. However, only a handful of studies have focused their efforts in analyzing the important relationship between survivin variants and adipokines [39, 46, 47].

We also investigated the potential correlation between the expression of *LEP*, *ADIPOQ*, and the three survivin variants in BCa, and whether the expression of these genes was significantly different between this last group and the BBT group. Overall, survivin has been suggested as a cancer biomarker [48], and regarding to BCa, it has also been associated with poor prognosis and suggested as a biomarker [40, 42]. Nevertheless, the general consensus is that no single molecule may be enough to serve as dictator of the presence or absence of any given cancer [3], even less so, if the molecule presents three different variants. Rather than focusing in a single molecule, the ultimate diagnosis method ought to include multiple biomarkers. In this matter, *LEP* and *ADIPOQ* have demonstrated to be important molecules. They both presented similar levels in BCa and BBT samples, suggesting that the underexpression observed in BCa may begin since a benign stage. Therefore, *LEP* and *ADIPOQ* expressions may be combined with those of survivin variants to potentially serve as BCa biomarkers.

The article "Altered Expression of Survivin Variants S-2B and S-WT in Breast Cancer Is Related to Adipokine Expression" was published in 2022. Journal: J Oncol.

It is important to remark that to the best our knowledge the relationship between these three survivin variants and the two adipokines has not been previously reported. Previous reports have focused solely on investigating the relationship between wild-type survivin and these adipokines; however, they have not specifically pointed out any of its three variants. Our study is the first to report a correlation between *LEP* and *ADIPOQ*, specifically with *S-2B* and *S-WT*. Likewise and very interestingly, although no correlation was found, we observed that in most samples with high *LEP* expression (stage IA), not quantifiable levels of *S-ΔEx3* were measured; however, this potentially negative correlation requires further investigation.

## 4. Conclusions

Here, we present evidence in the existing correlation between the expression of three different survivin variants and adipokines *LEP* and *ADIPOQ*, as well as their potential relationship with BCa development. Globally, higher *S-2B* and *S-WT* expressions were observed in patients with this pathology, whereas *S-ΔEx3* expression remained unaltered; however, the expression of *S-ΔEx3* statistically increased in advanced BCa stages. Moreover, *S-2B* and *S-WT* showed an important overexpression in high-aggressiveness BCa. Furthermore, our results demonstrated that not all survivin variants are correlated with *LEP* and *ADIPOQ*, as only *S-WT* and *S-2B* correlate with the expression of these two genes. It is important to further analyze the relationship of these genes to elucidate their complete implications in BCa development and to discover new biomarkers for this disease. Although so far has been proven complicated to diagnose cancer based on a single biomarker, the answer to this problem may recede not in one but in a set of biomarkers.

## Figures and Tables

**Figure 1:** Relative expression of *S-WT*, *S-2B*, *S-ΔEx3*, *LEP*, and *ADIPOQ*. Relative expression was compared between groups using the number of samples described for each gene in the result section. RT-qPCR exhibited significantly higher expression levels of *S-WT* and *S-2B* in BCa patients. Our results did not show a significant difference in the expression of *S-ΔEx3*, *LEP*, and *ADIPOQ* between groups. Bars represent mean values ± SD. ^∗∗^*p* < 0.01.

The article "Altered Expression of Survivin Variants S-2B and S-WT in Breast Cancer Is Related to Adipokine Expression" was published in 2022. Journal: J Oncol.

**Figure 2:** Relative expression of *S-WT*, *S-2B*, *S-ΔEx3*, *LEP*, and *ADIPOQ* in different BCa stages. Relative expression was compared among stages using the number of samples described for each gene in Table 2. Early stage patients exhibited the highest *LEP* expression (IA = 11.49), and late stage patients showed the lowest expression levels (IIIB = 0.05). On the other hand, we found the lowest *S-ΔEx3* expression in patients with low-grade tumors (IA = 0.14) and a gradual increase, until reaching the highest expression in stage IIIB (15.39). Bars represent mean values ± SD. ^∗^*p* < 0.05.

**Figure 3:** Relative expression of *S-WT*, *S-2B*, *S-ΔEx3*, *LEP*, and *ADIPOQ* in different BCa aggressiveness. Low-aggressiveness BCa subtypes luminal A, B, and HER2 are included in the luminal group, and high-aggressiveness BCa subtypes HER2-enriched and Basal-like are included in the HER2-basal group. Results showed a significant overexpression of *S-WT* and *S-2B* in high-aggressiveness BCa. Bars represent mean values ± SD. ^∗^*p* < 0.05.

**Figure 4:** Correlation analysis between relative expression of survivin variants and adipokines in BCa. A random correlation analysis was performed to our set of studied genes. Each data point represents a sample where both genes were present in quantifiable levels. *LEP* and *ADIPOQ* show a strong positive correlation closely to a coefficient of 1. Similarly, *S-2B* and *S-WT* display a strong positive correlation. Furthermore, although some were moderate, we observed correlations such as the negative relationship of *LEP* with *S-2B* and *S-WT* and the negative relationship of *ADIPOQ* and these same two survivin variants. Lastly, we did not observe a correlation between the expression of adipokines and *S-ΔEx3*.

**Table 1:** Clinicopathological characterization of BCa and BBT patients.

	BCa patients	BBT patients	*p* value
Age^a^	55.37 ± 14.45	40.75 ± 7.95	0.001^∗∗^
BMI^b^	27.66 ± 14.18	30.06 ± 6.13	0.14
Age of menarche^a^	13.41 ± 1.58	12.85 ± 1.46	0.223
Age of menopause^a^	47.43 ± 4.05	39.67 ± 6.12	0.010^∗^
Age of first pregnancy^a^	30.41 ± 6.40	20.44 ± 4.29	0.001^∗∗^
Number of pregnancies	4	2	0.138

Values represent mean ± SD. BCa: breast cancer; BTT: benign breast tumor. ^a^In years. ^b^In kg/m^2^. ^∗^*p* < 0.05; ^∗∗^*p* < 0.01.

**Table 2:** Number of samples per cancer stage for BCa group and gene.

Cancer stage	BCa group	S-WT	S-2B	S-*Δ*EX3	LEP	ADIPOQ
IA	3 (11.12)	3 (11.12)	3 (11.12)	1 (0.27)	3 (11.12)	3 (11.12)
IIA	9 (33.33)	9 (33.33)	8 (29.62)	6 (22.22)	9 (33.33)	9 (33.33)
IIB	6 (22.22)	5 (18.52)	4 (14.81)	3 (11.12)	5 (18.52)	5 (18.52)
IIIA	4 (14.81)	4 (14.81)	3 (11.12)	3 (11.12)	4 (14.81)	4 (14.81)
IIIB	5 (18.52)	4 (14.81)	2 (0.54)	2 (0.54)	4 (14.81)	4 (14.81)
Total	27 (100)	25 (91.33)^a^	20 (74.07)^a^	15 (55.55)^a^	25 (91.33)^a^	25 (91.33)^a^

Number in parenthesis represents the percentage as to the total of samples in the BCa group. BCa: breast cancer. ^a^Percentage of samples that presented quantifiable gene expression.

The article "Altered Expression of Survivin Variants S-2B and S-WT in Breast Cancer Is Related to Adipokine Expression" was published in 2022. Journal: J Oncol.

## Data Availability

Clinicopathological data presented in this work was the only information available in the hospital database. Raw data supporting our findings were generated at the Universidad Autonoma de Sinaloa and at the Universidad Politecnica de Sinaloa. Raw data is available if requested from the corresponding author.
